# Tualang Honey Protects against BPA-Induced Morphological Abnormalities and Disruption of ER*α*, ER*β*, and C3 mRNA and Protein Expressions in the Uterus of Rats

**DOI:** 10.1155/2015/202874

**Published:** 2015-12-14

**Authors:** Siti Sarah Mohamad Zaid, Normadiah M. Kassim, Shatrah Othman

**Affiliations:** ^1^Department of Anatomy, Faculty of Medicine, University of Malaya, 50603 Kuala Lumpur, Malaysia; ^2^Department of Environmental Sciences, Faculty of Environmental Studies, Universiti Putra Malaysia, 43400 Serdang, Selangor, Malaysia; ^3^Department of Molecular Medicine, Faculty of Medicine, University of Malaya, 50603 Kuala Lumpur, Malaysia

## Abstract

Bisphenol A (BPA) is an endocrine disrupting chemical (EDC) that can disrupt the normal functions of the reproductive system. The objective of the study is to investigate the potential protective effects of Tualang honey against BPA-induced uterine toxicity in pubertal rats. The rats were administered with BPA by oral gavage over a period of six weeks. Uterine toxicity in BPA-exposed rats was determined by the degree of the morphological abnormalities, increased lipid peroxidation, and dysregulated expression and distribution of ER*α*, ER*β*, and C3 as compared to the control rats. Concurrent treatment of rats with BPA and Tualang honey significantly improved the uterine morphological abnormalities, reduced lipid peroxidation, and normalized ER*α*, ER*β*, and C3 expressions and distribution. There were no abnormal changes observed in rats treated with Tualang honey alone, comparable with the control rats. In conclusion, Tualang honey has potential roles in protecting the uterus from BPA-induced toxicity, possibly accounted for by its phytochemical properties.

## 1. Introduction

Bisphenol A (BPA) (2,2-bis(4-hydroxyphenyl)) is one of the most ubiquitous environmental endocrine disrupting chemicals (EDC) in the world. It is widely used in industries as plasticizer for the production of polycarbonate plastics epoxy resins and as nonpolymer additive to other plastics [1]. It has received significant worldwide attention due to its exposure to human through leaches from the inner lining of food and beverage containers, plastic bottles, dental sealants, water supply pipes, and adhesives [2].

Many studies have revealed the negative effects of BPA on the development of the reproductive system in humans and laboratory animals [3, 4]. BPA has been detected in the serum and follicular and amniotic fluids [5], fetal serum [6], milk of nursing mothers [7], and urine [8, 9]. These reports suggest that humans are routinely exposed to BPA. Thus, it has fueled additional concern in human minds about BPA on their health.

Numerous studies have reported that BPA could induce morphological and functional alterations of the female genital system, particularly on the uterus [3, 10]. The main function of uterus is regulated by cyclic changes of sexual steroid hormones, and for this reason, it is widely used as a classical target organ to determine estrogenic effects of BPA [11]. BPA was shown to cause uterine disruptions by influencing the expression and distribution of estrogen receptor-*α* (ER*α*) and estrogen receptor-*β* (ER*β*) [12]. BPA was also reported to reduce uterine immunity via dysregulation of complement C3 expression that caused ascending infections in the female reproductive tract [13]. Study by Xiao et al. (2011) has found that prenatal exposure to BPA could adversely affect transportation and preimplantation of the embryo from disturbance in the uterine receptivity that lead to infertility in female rats [14]. Furthermore, BPA has been reported to promote oxidative stress and inflammation in the female reproductive tract which might contribute to the morphological and functional abnormalities [15].

Natural compounds with antioxidant properties have been extensively studied as a means to counter disease-associated oxidative stress [16]. With these concerns in mind, we used a natural product with high antioxidant content, namely, Tualang honey (Agromas, Malaysia) as a possible potential therapeutic agent to counter the deleterious effects of BPA. Previous scientific studies have claimed that Tualang honey has the capability to ameliorate oxidative stress in renal and pancreas of streptozotocin-induced diabetic rats [17], reverse atrophic uterus and vagina [18], and to improve osteoporotic bone [19] in postmenopausal animal model. In addition, Tualang honey has the capability to protect against cigarette-induced damage on testis [20] and to counter the proliferation of oral squamous cell carcinomas (OSCC) [21], human osteosarcoma [21], and keloid fibroblasts [22].

Tualang honey, a dark brownish honey has been reported to contain more than 200 substances including sugars, amino acids, vitamins, minerals, enzymes, organic acids, and phytochemicals. The primary content of Tualang honey is inverted sugars that consist of fructose 29.6%, glucose 30%, sucrose 0.6%, and maltose 7.9% as well as a small amount of complex mixture of other saccharides (disaccharides, trisaccharides, and oligosaccharides) [23]. It also contains high total phenolic compounds (gallic, syringic, benzoic, trans-cinnamic, p-coumaric, and caffeic acids) and flavonoids (catechin, kaempferol, naringenin, luteolin, and apigenin) [24]. It has tremendous antioxidant properties with high radical scavenging and antioxidant activities [25]. The other compounds present in Tualang honey are stearic acids, furfural, acetic acid, 2-furylmethylketone, palmitic acid, ethyl linoleate, oleic acid, 2-hyroxy-2-cyclopenten-1-one, hyacinthine, and 5-methyl furfural [23].

The aims of our study were to investigate the effects of subchronic administration of BPA on the uterine morphology and function by determining the lipid peroxidation, protein distribution, and mRNA expressions of estrogen receptor-*α*, estrogen receptor-*β*, and complement C3. Consequently, investigation of the possible protective effects of Tualang honey against BPA-induced uterine toxicity is executed.

## 2. Material and Methods

### 2.1. Tualang Honey (Agromas, Malaysia)

Tualang honey was purchased from the Federal Agricultural Marketing Authority (FAMA), under the Ministry of Agriculture and Agro-Based Industry, Malaysia. Tualang honey is wild multifloral honey collected from* Apis dorsata's* beehive that is built on a giant tree,* Koompassia excelsa* (locally known as Tualang tree), in the rain forest of Kedah, Malaysia. At Honey Processing Centre in Kuala Nerang, Kedah, the honey was processed through several stages (quality inspection, dehydration, packaging, and labeling). In brief, the honey was filtered to remove solid particles, concentrated in an oven at 40°C, and subjected to *γ* irradiation at 25 kGy at Sterilgamma (M) Sdn. Bhd. (Selangor, Malaysia). The water concentration of the honey was standardized by FAMA at 18%.

### 2.2. Animal Model and Experimental Design

Female Sprague rats (P21) were obtained from the Animal Husbandry, Faculty of Medicine, University of Malaya. All the experimental design and procedures were conducted according to the National Institutes of Health guide for the care and use of Laboratory animals (NIH Publications number 8023, revised 1978) which has been approved by the Animal Care and Committee (ACUC) of the University of Malaya. Throughout the experimental period, the rats were maintained under the standard laboratory conditions (temperature 25 ± 2°C, 50 ± 15% relative humidity, and normal photoperiod of 12 h dark and 12 h light) and supplied* ad libitum* with water and commercial pellet diet (Gold Coin Feedmills Pte. Ltd., Malaysia). The rats were placed in stainless steel cages with wood bedding and water was supplied in glass bottles to minimize additional exposures endocrine disruptors. They were acclimatized to the laboratory environment for seven days prior to the commencement of the experiment. At 28 days of age, the rats were randomly divided into four groups (*n* = 8 in each group).

NC group (negative control) was administered with the vehicle (0.2 mL of corn oil). PC group (positive control) was administered with BPA (10 mg/kg body weight suspended in corn oil). THC group (Tualang honey control) was administered with Tualang honey (200 mg/kg body weight 30 min before administration of corn oil). TH group (Tualang honey + BPA) was administered with Tualang honey (200 mg/kg body weight 30 min before administration of BPA at 10 mg/kg body weight). The procedure was performed in the morning (between 09:00 and 10:00 AM) once daily by oral gavage (to mimic the most likely route of human exposure) for six consecutive weeks. Throughout the administration period, daily body weight was recorded. After the last treatment, the rats were sacrificed during their diestrous phase.

Once the rat was sacrificed, the wet weight of the whole uterus was recorded for uterotrophic response evaluation. The left horn of the uterus was immediately fixed in 10% buffered formalin for histopathological analysis. One half of the right horn of uterus was kept in phosphate buffer for malondialdehyde (MDA) determination while the other half was kept in RNAlater for mRNA extraction and subsequently stored in −80°C freezer until further analysis. The dose selection of BPA at 10 mg/g body weight was based on previous studies where BPA at this dose was reported to induce disruption on the morphological and biochemical parameters in the reproductive system [3, 26–28]. As for Tualang honey, it was freshly prepared daily to avoid oxidation of the antioxidants content. The dose of Tualang honey at 200 mg/kg body weight was based on previous study that showed positive biological effects on female reproductive organs and the dose was equal to one tablespoon which is routinely taken by an adult human [18].

### 2.3. Histopathological Evaluation

The uteri were fixed in 10% buffered formalin for 24 hours prior to further processing for histopathological examination. The uteri were trimmed accordingly, dehydrated through a graded series of increasing concentration of ethanol, cleared in xylene, and finally embedded in paraffin to form paraffin block. Subsequently, tissue sections of 5 *μ*m thicknesses were obtained and mounted onto glass slides, deparaffinized in xylene, hydrated with water, and stained with hematoxylin and eosin (Sigma-Aldrich, USA). Once again, sections were dehydrated in a graded series of ethanol, cleared in xylene, and mounted with Canada Balsam (Sigma-Aldrich). All sections were analyzed for any morphological changes under a light microscope (Olympus CH-B145-2) attached to an image analyzer (NIS-Elements Advanced Research, Nikon, Japan). Representative micrographs were taken for future reference.

### 2.4. Histomorphometry

For histomorphometric analysis of the uterus, the tissue sections were reviewed and the clearest representative sections on each slide were photographed at ×20 and ×40 magnifications. The mean values of height of the luminal epithelial cells, thickness of the endometrium, and the myometrium layers were measured in six randomly chosen areas of the sections. All measurements (in *μ*m) were manually determined by tracing the on-screen images using a computer-image analyzing program (NIS-Elements Advanced Research, Nikon, Japan).

### 2.5. Immunohistochemistry

#### 2.5.1. Estrogen Receptor-*α* and Complement C3

The distribution of estrogen receptor-*α* and complement C3 in rat uteri was evaluated using ImmunoCruz Rabbit ABC staining system sc-2018 kit and ImmunoCruz Goat ABC staining system sc-2023 kit, respectively.

Briefly, tissue sections were deparaffinized, hydrated to water, boiled in 0.1 M sodium citrate buffer (pH 6.0) for 15 minutes, and incubated with 0.1%–1% of hydrogen peroxide for 10 minutes to quench the endogenous peroxidase activity. Nonspecific staining was blocked by incubating it in 1.5% blocking serum. Subsequently, the sections were incubated with primary antibody at 1 : 100 dilution of ER*α* (MC-20:sc-542, Santa Cruz Biotechnology, USA) or 1 : 100 dilution of C3 (V-20:sc-14612, Santa Cruz Biotechnology, USA) overnight at 4°C. On the following day, the sections were incubated with biotinylated secondary antibody for one hour and then incubated with AB enzyme reagent for another 30 minutes. Positive staining appeared (bluish in color) after incubation with peroxidase abstract for 10 minutes and, finally, the sections were counterstained with hematoxylin. The sections were then dehydrated through a graded series of ethanol, cleared in xylene and mounted with Canada Balsam (Sigma-Aldrich), and covered with glass coverslips before examination under light microscopy. The negative control tissue (not incubated with primary antibody) was included to ensure no false positive staining and for accurate interpretation of the staining results.

#### 2.5.2. Estrogen Receptor-*β*

The distribution of estrogen receptor-*β* in uterus rats was evaluated using Rabbit Specific HRP/DAB (ABC) Detection IHC Abcam kit.

Briefly, the sections were deparaffinized, hydrated, boiled in 0.1 M sodium citrate buffer (pH 6.0) for 15 minutes, and incubated with hydrogen peroxide for 20 minutes to quench the endogenous peroxidase activity. Nonspecific staining was blocked by incubation in protein block. Subsequently, the sections were incubated with primary antibody at 1 : 200 dilution (ER*β* antibody ab3576, Abcam, USA) overnight at 4°C. Next day, the sections were incubated with biotinylated secondary goat anti-polyvalent antibody for 30 minutes at room temperature. Positive staining developed after the incubation with DAB chromogen for 10 minutes, followed by counterstaining with haematoxylin. The sections were dehydrated in 2x 95% of ethanol, 2x 100%, and 3x xylenes for 10 seconds each. Finally, the sections were mounted with Canada Balsam (Sigma-Aldrich) and covered with glass coverslips for observation under light microscopy. The negative control tissue (not incubated with primary antibody) was included to ensure no false positive staining and accurate interpretation of the staining results.

#### 2.5.3. Determination of Malondialdehyde (MDA) Levels

MDA levels of uterus were measured by the double heating method [29] using Thiobarbituric Acid Reactive Substances (TBARS) assay (OxiSelect TBARS assay kit, Cell Biolabs, USA). The uterus of each animal was homogenized in phosphate buffered saline (PBS) containing butylated hydroxytoluene (BHT). Subsequently, the uterine homogenate was centrifuged at 10,000 g for 5 minutes to collect the supernatant for the TBARS assay.

Briefly, 100 *μ*L of samples and standards was mixed with 100 *μ*L of SDS lysis solution in appropriate tubes and incubated for 5 minutes at room temperature. Then, 250 *μ*L of TBA reagent was added to each tube followed by 60 minutes of incubation at 95°C. The tubes were cooled at room temperature in ice bath for five minutes. All the tubes were centrifuged at 3000 rpm for 15 minutes and 200 *μ*L of the supernatant was transferred to a 96-well microplate for measurement of absorbance using a spectrophotometer at 532 nm wavelength. The concentration of MDA was calculated using the absorbance coefficient of the MDA-TBA complex and expressed as micromoles per microgram protein (*μ*M/*μ*g protein).

### 2.6. mRNA Expression of ER*α*, ER*β*, and Complement C3

#### 2.6.1. Purification of Total RNA

Purification of total RNA of uterus was performed using RNeasy Protect Mini Kit, Qiagen, USA. 30 mg of tissue samples of uteri was disrupted and homogenized in Buffer RLT. The lysate was centrifuged at maximum speed (12000 rpm). The supernatant were transferred into a new 1.5 mL tube and one volume of 70% of ethanol was added. This sample was transferred into an RNeasy spin column and centrifuged and the flow-through was discarded. Subsequently, buffer RPE was added to the RNeasy spin column and centrifuged for one minute at 10000 rpm and the flow-through was again discarded. This step was repeated but centrifugation was performed for a longer period of two minutes.

Finally, the spin column was placed in a new 1.5 mL tube, added with 30 *μ*L of RNase-free water, and centrifuged at 10000 rpm for one minute to elute the RNA. Finally, measurement of the concentration and purity of RNA was done by using a NanoDrop (BioTek, USA) at OD_260/280_ while the quality assessment was performed via denaturing agarose gel electrophoresis. The RNA was kept at −20°C until further analysis.

#### 2.6.2. Reverse Transcription of RNA to cDNA

Reverse transcription (RT) of RNA to single-stranded cDNA was done using the Applied Biosystems Kit, USA. Equal amounts of RNA (300 ng) from each sample were reverse-transcribed into cDNA. Each RT reaction mix consisted of 2x RT buffer (10 *μ*L), 1 *μ*L of reverse transcriptase, nuclease-free water, and RNA sample made up to a total volume of 20 *μ*L. The reaction mixes were briefly centrifuged to spin down the contents and eliminate air bubbles. Finally, the tubes were placed in a programmed thermal cycler (Thermo Scientific) for 60 minutes at 37°C followed by five minutes at 95°C.

#### 2.6.3. Quantitative Real-Time PCR of Selected Genes

Quantitative real-time PCR of selected genes was carried out using Applied Biosystems Kit, USA. The PCR reaction mix (reaction size of 20 *μ*L) was prepared in triplicate. Each PCR reaction mix consists of 20x TaqMan Gene Expression Assay (1 *μ*L), 2x TaqMan Gene Expression Master Mix (10 *μ*L), cDNA template (4 *μ*L), and RNase-free water (5 *μ*L). The endogenous control gene used in this study was *β*-actin mRNA. In order to ensure specific amplification, three types of controls (water only, reaction without primers, and templates derived without reverse transcriptase) were included in the PCR reaction. The prepared PCR reaction mix was inverted to mix the reaction components, followed by brief centrifugation. Twenty *μ*L of PCR reaction mix was transfer to each appropriate 96-well reaction plate and briefly centrifuged.

Finally, the plate was placed in the StepOne Plus Real-Time PCR system (Applied Biosystems, USA), followed by automated amplification of the genes of interest. The point at which exponential amplification of the PCR products begins (values for cycle threshold: CT) was determined using the Applied Biosystems software. Relative abundances of the target mRNA were calculated using the 2^−ΔΔCT^ method [30]. The experiment was repeated three times to ensure the validity of the results. The relative mRNA expression levels for each selected gene were calculated in terms of the *β*-actin internal control. The sequences of primer used for the amplification of gene are shown in Table 1.

### 2.7. Statistical Analysis

All statistical evaluations were performed with Statistical Package for Social Sciences (SPSS Inc. Chicago, Illinois, USA, version 18.0 for Windows). Firstly, Shapiro-Wilk *W* test was performed to test whether all results followed a normal distribution (normally distributed if *P* value was greater than 0.05). Parametric variables were analyzed using One-way analysis of variance (ANOVA) followed by Bonferroni test for multiple comparisons to identify significant differences between groups. Values were reported as Mean ± SEM. *P* < 0.05 was considered significant.

## 3. Results

### 3.1. Body Weight and Uterine Weight

In toxicological studies, analysis of body weight and the weight of selected organs is a sensitive indicator for adverse effects of chemical exposure. In particular, analysis of normalization of absolute organ weight to body weight (relative organ weight) is a more accurate analytical endpoint for the identification of harmful effects of a toxic agent on the organ weights. The changes in body weight gain and uterine relative weight of animals in all experimental groups are shown in Table 2 and Figures 1(a) and 1(b), respectively.

To determine whether BPA exposure induces changes in body weight as a result of toxicity effects, the body weight of all rats was monitored throughout the experimental period. Although changes in the body weight gain were not statistically significant between BPA-exposed group and all the other groups, six weeks of subchronic exposure to BPA in the PC group had caused a slight increment (17.3%) in the body weight gain compared to the control animals (NC group). Similar increment (16.55%) in body weight gain was also noted in rats concurrently treated with BPA and Tualang honey (TH group). The changes in body weight gain for Tualang honey treated alone (THC group) rats were comparable to the control rats (NC group).

Similarly, the changes in uterine weight were recorded at the end of the administration period since this could be used as an indicator for any changes in the normal functions. After six weeks of BPA exposure (PC group), significant decline was observed in the uterine relative weight by 25% compared to the control rats (NC group). However, concurrent treatment of rats with BPA and Tualang honey (TH group) had significantly prevented this effect. The uterine relative weight in rats treated with Tualang honey alone (THC group) was comparable to the control rat (NC group), reflecting that Tualang honey itself has no deleterious effect on the uterus weight.

### 3.2. Malondialdehyde (MDA) Level

Lipid peroxides are unstable primary products of lipid peroxidation which decompose to the stable form malondialdehyde (MDA). Measurement of the MDA levels as the end product of lipid peroxidation is a widely accepted assay and is considered to be a crucial index of oxidative stress associated with organ pathophysiology in animals.

As shown in Table 2 and Figure 2, a significant increase in the MDA level by 49.7% was noted in rats exposed to BPA (PC group) as compared to the control rats (NC group). However, concurrent treatment of BPA with Tualang honey had led to significant reduction in the MDA levels (TH group). The MDA level was not affected by Tualang honey treatment alone (THC group) and the value is comparable to the normal rats (NC group).

### 3.3. Uterine Histomorphometry Analysis

As shown in Table 2 and Figures 3(a), 3(b), and 3(c), BPA exposure had caused a significant reduction in all histomorphometric parameters (including luminal epithelial cells and thickness of the endometrium and myometrium layers) (PC group) when compared to all the other groups (NC, TH, and THC groups).

In the BPA-exposed rats (PC group), the reductions were to 38.11%, 14.88%, and 23.66% in luminal epithelial cells height and endometrial and myometrial thickness, respectively. Interestingly, consistent with the reduction of the uterine relative weight, concurrent treatment of rats with BPA and Tualang honey (TH group) significantly prevented the reduction in these parameters. Meanwhile, the values of these parameters in the three groups were comparable to each other.

### 3.4. Morphology of the Uterus

Morphological analysis of the representative uteri from sections of all groups is shown in Figure 4. The morphological changes were consistent with the histomorphometric analysis.

In the control rats (NC group), normal histological appearance was observed (Figures 4(A), 4(B), and 4(C)). The luminal epithelial cells were made up of tall pseudostratified columnar epithelium, cylindrical in shape with well-rounded nuclei, and rested on a prominent basement membrane. The lamina propria was intact with healthy endometrial glands and high cellular content in the stroma. A number of mitotic figures were visible in glandular epithelial cells. The myometrium appeared to be normal. The histological appearances of the endometria in rats treated with Tualang honey alone (THC group) were comparable to the control rats (NC group) (Figures 4(G), 4(H), and 4(I)).

The uterus of BPA-exposed rats (PC group) exhibited disruptive changes as shown in Figures 4(D), 4(E), and 4(F), when compared to the control rats (NC group). The luminal epithelial cells were shorter, the stroma had less cell population and appeared disorganized, and some cells were distorted and had irregular-shaped nuclei. Some of the nuclei had more condensed chromatin. There were very little interstitial intracellular spaces between the stroma cells. The endometrial glands appeared unhealthy by being smaller in size and lined by shrunken and distorted epithelial cells with irregularly shaped nuclei and some pyknotic nuclei, which are less organized and reduced in number. The smooth muscle bundles of the myometrium which were also seen smaller and shrunken with the organizations of the inner circular and outer longitudinal smooth muscle fibers looked disintegrated.

In comparison with BPA-exposed rats (PC group), the uterine morphology of the Tualang honey (TH group) (Figures 4(J), 4(K), and 4(L)) showed slightly improved surface epithelium, but had healthy looking stromal cell population with larger stromal cells and relatively more interstitial spaces between cells compared to the PC group. The endometrial glands looked normal, lined by glandular epithelium, very much comparable to the NC group. Moreover, the myometrium also appeared normal.

### 3.5. ER*α*, ER*β*, and C3 Protein Distribution

The representative uterine tissue sections were stained using immunohistochemical technique to evaluate cell specific changes in the ER*α*, ER*β*, and complement C3 proteins. These proteins are localized in the nuclei of epithelial and stromal cells of the uterus.

In general, the staining intensity of ER*α* protein receptor expression in all representative uterine sections was highest in the luminal and glandular epithelial cells but lower staining intensity was found in the cells of endometrial stroma (about 50 to 80%) (Figure 5). Among all groups, the most pronounced immunostaining intensity was observed in the control rats (NC groups) (Figures 5(C) and 5(D)) and the Tualang honey alone treated rats (THC group) (Figures 5(G) and 5(H)). As expected, lower immunostaining intensity was observed in BPA-exposed rats (PC group) (Figures 5(E) and 5(F)) and in rats with concurrent treatment with Tualang honey (TH group) (Figures 5(I) and 5(J)).

As shown in Figure 6, the immunostaining patterns and intensities of ER*β* were different from the ER*α*. Comparable immunostaining intensities were observed in rats of NC group (Figures 6(C) and 6(D)), THC group (Figures 6(G) and 6 (H)), and TH group (Figures 6(I) and 6(J)), while there was less immunostaining intensity in all compartments (namely, luminal and glandular epithelial cells and stroma) in the BPA-exposed rats (PC group).

For complement C3 protein expression, the immunostaining intensity was highest in both the control rats (NC group) and Tualang honey alone treated rats (THC group) (Figures 7(C), 7(D) and 7(G), 7(H), resp.). There was less immunostaining intensity in the BPA-exposed rats (PC group) (Figures 7(E) and 7(F)) while there was slightly higher intensity of staining in the stroma of rats with concurrent treatment with Tualang honey (TH group) (Figures 7(I) and 7(J)).

### 3.6. ER*α*, ER*β*, and C3 mRNA Expression

The changes in mRNA expression of estrogen-related genes were measured to support the immunohistochemistry analysis. The ER*α*, ER*β*, and complement C3 mRNA expression are shown in Figures 8(a), 8(b), and 8(c).

As shown in Figure 8(a), BPA exposure in PC group animals significantly downregulated the ER*α* mRNA expression by approximately 4-fold as compared to the control rats (NC group). However, the magnitude was reduced to 3-fold by concurrent treatment with Tualang honey (TH group). In contrast, treatment with Tualang honey (THC group) showed 1.5-fold induction in the ER*α* mRNA expression compared to the control group.

Figure 8(b) shows a dissimilar pattern of ER*β* mRNA expression compared to ER*α* mRNA expression. As compared to the control rats (NC group), the expression of ER*β* was significantly upregulated by approximately 1.4-fold in BPA-exposed rats (PC group) and this was reduced to 1.1-fold by concurrent treatment of Tualang honey (TH group). This indicates that concurrent treatment with Tualang honey was able to reduce the ER*β* mRNA expression in BPA-exposed rats by 80%. Meanwhile, Tualang honey alone (THC group) had no effect on the ER*β* mRNA expression with the value of expression comparable to the control rats (NC group).

As shown in Figure 8(c), BPA exposure (PC group) caused dramatic suppression of the complement C3 mRNA expression by almost 90% as compared to the control rats (NC group). Surprisingly, this effect was completely reversed with concurrent treatment with Tualang honey (TH group). In fact, the C3 mRNA expression in the Tualang honey group (TH group) was 1.8-fold higher than the control rats (NC group). Tualang honey alone had no effect on the C3 mRNA expression with the value of expression comparable to the control rats (NC group).

## 4. Discussion

BPA, as an endocrine disrupting chemical (EDC), has the capability to mimic, enhance, or inhibit the activity of natural estrogen and to disrupt the functions of estrogen nuclear hormone receptors in a diverse set of target tissues [8, 13, 15, 34]. Thus, exclusively defining BPA as an environmental estrogen or selective estrogen receptor modulator (SERM) is indeed inaccurate [2].

In the last few decades, a considerable amount of evidence has been accumulated which demonstrates the fact that young women may be at high risk of reproductive infertility due to continuous exposure to numerous BPA products in their daily lives [35]. With this concern in mind, our present study had investigated the disruptive effects of BPA on the female reproductive physiology with special reference to the morphology, oxidative markers, and protein and molecular changes that occur in the rat uterus. In addition, the potential protective roles of Tualang honey as a natural product in reducing the disruptive effects of BPA on the above-mentioned selected parameters were evaluated. The mechanisms of the translational and transcription factors in estrogen receptors were also investigated. In addition to the classical* in vivo* tool (uterotrophic assay), more sensitive tools such as the analysis of gene transcription and protein expression were adopted to investigate the molecular responses due to BPA exposure.

In toxicology study, the differences in body and organ weights between untreated and treated animals can be a reliable indicator for the toxicity effects of the test compounds [36]. In the present study, the toxicology data showed that the effects of BPA appear to be very specific to the uterus as the reduction in weight seems to affect the uterus itself, without having significant effects on the whole body weight. These current results are in agreement with a previous report by Ashby et al. [37]. In contrast, others have shown that BPA exposure in rodent animals was reported to be associated with weight gain [38–40].

BPA is one of the suggested EDCs that induce reactive oxygen species (ROS) that play important roles in the pathology of female reproductive diseases such as uterine endometriosis [35]. Furthermore, lipid peroxidation (LPO) is a process of interaction between reactive oxygen species (ROS) and the cellular membrane that induces damage to cellular macromolecules and DNA [41]. Since malondialdehyde (MDA) is a secondary product of LPO, it is generally accepted as an oxidative stress marker [42]. The relationship between oxidative stress and infertility among women has been proven in several scientific studies [43, 44]. Epidemiological data showed that higher levels of reactive oxygen species (ROS) and lower antioxidant levels were detected in infertile women compared to fertile women [45, 46]. In the present study, the uterine MDA level in BPA-exposed animals was significantly higher compared to the normal control animals. The results could be due to lipid peroxidation process by BPA and this result correlated well with the histopathological, immunohistochemical, and gene expression analyses.

Treatment with Tualang honey in BPA-exposed rats significantly reduced the uterine MDA levels. This observation could be due to the antioxidant effects of Tualang honey which cause reduction in the number of free radicals. This explanation is based on several published data that reported Tualang honey as an effective antioxidant in reducing the MDA levels in human subjects and animal models [17, 47].

In addition to that, striking morphologic changes of the uterus (disruption of the normal structure of the luminal epithelium, endometrium, myometrium, and glandular epithelial cells) associated with oxidative stress were apparent in BPA-exposed rats compared to the controls. These morphological changes could be related to the potential direct actions of BPA on the DNA itself that results in alteration of gene expression. BPA-induced DNA damage has been evidently reported, in both* in vivo* and* in vitro* studies [48, 49]. This is because BPA can be oxidized to bisphenol-o-quinone that covalently binds to deoxyguanosine to form DNA adducts. Subsequently, DNA adducts cause improper and incomplete replication that leads to the formation of atypical cells.

Interestingly, the disruptive effects of BPA on the uterine morphology were partially reduced following concurrent treatment with Tualang honey. The improvement could be, again, accounted for by the high natural antioxidant contents in Tualang honey in addition to the carbohydrates, amino acids, proteins, organic acids, vitamins, and various phytochemicals [24, 50]. In the natural state, cells of our body are capable of maintaining the normal equilibrium of antioxidant-oxidative stress balance by neutralizing or directly diminishing the oxidative damage by means of enzymatic and nonenzymatic antioxidants [51]. Evidently, Tualang honey contains nonenzymatic antioxidants such as vitamins E and C with their interactive effects as lipophilic and hydrophilic free-radical scavengers, respectively [52] hence possibly explaining the improvement observed in treated rats.

Vitamin E resides mainly in the cell membranes, thus playing an important role in the maintenance of cell membranes [53]. Meanwhile, the major function of vitamin C is as a scavenger of free radicals in the extracellular fluid, deceiving radicals in the aqueous phase, protecting biomembranes from peroxidase impairment, and regenerating tocopherol (vitamin E) from tocopheroxyl radicals in the membrane [54]. Several studies have found that both antioxidants can mitigate adverse pathological impacts by minimizing the genotoxicity and cytotoxicity effects in the cells [55–57]. Flavonols (quercetin and kaempferol) with weak estrogenic activities are attributed to the decrease in the intracellular reactive oxygen species (ROS) by a mechanism that involves estrogen receptors [58]. Thus, in our study, the antioxidant properties of Tualang honey could be contributing to the protective effects in cells by trapping and inactivating of free radicals as observed in the improvement of the heterogeneous cell types of the uterus (stromal, luminal epithelium, endometrial glands, and smooth muscle).

Nonetheless, the morphological recovery following treatment with Tualang honey in BPA-exposed uterus seems to be partial. This may be due to the presence of other reactive oxygen species that could also be in play to cause the disruptive effects. Moreover, even after removal of BPA, the inactive detoxifying proteins/enzymes may require a certain period of time to recover, as supported by Chevallet et al. [59].

Other findings in our study which are also in line with previous studies showed that BPA can disrupt the development, growth, and functions of the uterus by interrupting the regulation of mRNA expression and protein distribution of ER*α*, ER*β*, and complement C3 [12, 13, 60]. Estrogen receptor (ER) is a member of steroid receptor superfamily, a ligand-activated enhancer protein that is activated by the hormone estrogen (17*β*-estradiol) and is able to regulate gene transcription via estrogen responsive elements [61]. Unfortunately, it can also be activated by other compounds including endocrine disrupting chemical such as BPA [62]. The ER is encoded by two subtype genes, namely, ER*α* and ER*β*, that function as a signal transducer and a transcription factor in modulating the expression of target genes [63]. The endogenous estrogen (17*β*-estradiol) has a lower binding affinity to ER*β* than ER*α* [34] but both receptors share similarity in terms of transactivation via estrogen responsive element (ERE) [64]. In contrast, they possess dissimilar functions with regard to their roles in transcription activation, which depend very much on the ligands and their responsive elements [65].

BPA is considered weak environmental estrogen since its binding affinity to ER*α* and ER*β* is estimated to be 10,000-fold lower than the endogenous estrogen, with a relative binding affinity of 6-fold higher in ER*β* compared to ER*α* [34, 62]. On the other hand, in some cell types, BPA exhibits estradiol-like agonist activity via ER*β* and a mixed agonist/antagonist activity via ER*α* [15]. Both subtypes contain a ligand-dependent transactivation domain, named AF2 (Activation Function 2), for activation of transcription of target genes by the recruitment of transcriptional cofactors steroid receptor coactivator-1 (SRC-1) and transcriptional intermediary factor-2 (TIF-2) [66]. The disruptive role of BPA in this pathway significantly increases the recruitment of these cofactors [67]. This could be a possible explanation for our present data that showed significant upregulation in the expression of mRNA and higher protein distribution of ER*β* in BPA-exposed animals (PC group) as compared to the control rats.

In our study, besides the role of lipid peroxidation, the upregulation of ER*β* in BPA-exposed animals could be attributed to the disruptive effects in the uterus. A report in 2000 by Weihua et al. revealed that, in the uterus, ER*β* acts as a modulator of ER*α*-mediated gene transcription [68]. The role of ER*β* is as a transdominant repressor that inhibits the ER*α* transcriptional activity [69]. The inhibitory effects are due to the ability of ER*β* to form heterodimers with ER*α*, which in turn regulate the functions of estrogen receptors [70]. Thus, unlike ER*α*, ER*β* does not have classic uterotrophic effects but rather disruptive effects on ER*α*.

Other studies via crystallography structure analysis and computer modeling studies have found that BPA has higher binding affinity to ERR*γ* to ER*α* [71, 72]. ERR*γ* is an orphan nuclear receptor that belongs to the ERR family (estrogen receptor-related) [73]. Although both ER*α* and ERR*γ* receptors share similar sequence homology, 17*β*-estradiol does not associate to ERR*γ* [74]. The BPA-ERR*γ* interaction was suggested to trigger heterodimerization between ER*α* and ERR*γ* which results in suppression of the transcriptional activity of the ER*α* [71]. Similarly, Huppunen and Aarnisalo also reported that the modulation of BPA as an inhibitor on ER*α* signaling is also via ERR*γ* [75]. Such interaction could be an explanation for our present data that showed significant downregulation of mRNA expression and lower protein distribution of ER*α* in BPA-exposed animals (PC group) compared to the control normal animals. In addition, the ER*α* mRNA expression was also significantly higher in Tualang honey treated rats. However, the protein distribution did not differ much from the normal control rats. Hence, these results suggest that Tualang honey is likely to modulate the ER*α* mRNA expression at the transcriptional level but not at the translational level.

Complement C3 is involved in innate immunity. The crucial role of C3 is to regulate any activation of host cell damage by promoting phagocytosis, initiating local inflammatory responses against pathogens, and to instruct appropriate adaptive immune response towards antigens for a humoral response [76]. In 2004, Seidlová-Wuttke et al. have used quantitative RT-PCR analysis to investigate the effects of BPA on C3 mRNA transcription in rat uterus [13]. According to the authors, estradiol treatment significantly upregulated the C3 mRNA expression. Interestingly, the effect was not mimicked by BPA exposure where downregulation of C3 mRNA expression was observed. This effect was also observed in our present study. However, concurrent treatment with Tualang honey was able to significantly increase the C3 expression, indicating some improvement in the innate immune system. Interestingly, the mRNA expression in Tualang honey treated rats was also significantly higher compared to the control animals. This could be due to higher activation of transcriptional activity C3 induced by certain bioactive compounds that oppose the disturbance effects of BPA on the innate immune system. However, the protein distribution in Tualang honey treated rats did not differ much from the BPA-exposed rats. Hence, these results suggest that Tualang honey is likely to modulate the C3 mRNA expression at the transcriptional level but not at the translational level.

The improvements of protein and molecular levels of ER*α*, ER*β*, and C3 in BPA-exposed animals treated by Tualang honey could be explained by the fact that Tualang honey contains high nutritional profile antioxidants including flavonoids, specifically flavonols [58]. The two main naturally occurring flavonols, namely, quercetin and kaempferol share structural similarities with 17*β*-estradiol and hence may potentially have weak estrogenic effects [58]. Evidence from our previous study have shown that besides the ability to scavenge oxidants and free radicals [19], biologically active estrogen-like compounds in Tualang honey also improved the atrophy state of uterus and vagina [18]. In addition, our previous findings also found that the potential competitive binding of these compounds also contributed to the improvement of the hypothalamic-pituitary axis function in BPA-exposed animals [77] as also supported by an earlier study [78].

The effects of lipid peroxidation of BPA on DNA damage have also been extensively tested in* in vivo* and* in vitro* studies [79–81]. The antigenotoxicity effects of Tualang honey were reported to occur via several mechanisms: the upregulation of double stranded DNA repair enzymes [82], reduction of cyclobutane pyrimidine dimers and 8-oxo-dG-positive cells (biomarkers of DNA damage) [83], and induction of apoptosis [84]. Similar protective mechanisms against DNA damage have been suggested in studies on Buckwheat honey and honey from arid regions that are also in line with the current Tualang honey findings [85, 86].

## 5. Conclusions

In conclusion, Tualang honey has potential roles in reducing BPA-induced uterine disruption, possibly accounted for by its phytochemical properties. In view of this, Tualang honey could be suggested as a promising natural product candidate in reducing the toxicity effects of BPA in the uterus. Thus, further investigation is warranted to establish precise and better understanding of the roles of phytochemical compounds in Tualang honey that account for the reduction in BPA-induced uterine toxicity.

## Figures and Tables

**Figure 1:** (a) Changes in body weight gain. Body weight gains were not statistically different among all experimental groups. (b) Uteri relative weights in all experimental groups. BPA exposure which caused a significant decline in body weight was observed (PC group), while concurrent treatment of BPA with Tualang honey (TH group) significantly prevented the reduction in the relative body weight. Data are expressed as Mean ± SEM. (1) ^aaa^ *P* < 0.001 versus NC (negative control). (2) ^b^ *P* < 0.05, ^bb^ *P* < 0.01, and ^bbb^ *P* < 0.001 versus PC (BPA 10 mg/kg). (3) ^c^ *P* < 0.05 versus TH (Tualang honey 200 mg/kg + BPA 10 mg/kg). (4) ^dd^ *P* < 0.01 versus THC (Tualang honey 200 mg/kg).

**Figure 2:** Levels of malondialdehyde (MDA) in all experimental groups. Malondialdehyde level was significantly increased in BPA-exposed rats (PC group), while concurrent treatment of BPA with Tualang honey (TH group) has significantly prevented the increment effect of BPA. Data are expressed as Mean ± SEM. (1) ^aaa^ *P* < 0.001 versus NC (negative control). (2) ^b^ *P* < 0.05, ^bbb^ *P* < 0.001 versus PC (BPA 10 mg/kg). (3) ^c^ *P* < 0.05 versus TH (Tualang honey 200 mg/kg + BPA 10 mg/kg). (4) ^ddd^ *P* < 0.001 versus THC (Tualang honey 200 mg/kg).

**Figure 3:** (a) Height of luminal epithelial cells of uterus in all experimental groups. BPA-induced reduction in luminal epithelial height (PC group) was significantly prevented by concurrent treatment with Tualang honey (TH group). Data are expressed as Mean ± SEM. (1) ^a^ *P* < 0.05 and ^aaa^ *P* < 0.001 versus NC (negative control). (2) ^bbb^ *P* < 0.001 versus PC (BPA 10 mg/kg). (3) ^c^ *P* < 0.05 and ^cc^ *P* < 0.01 versus TH (Tualang honey 200 mg/kg + BPA 10 mg/kg). (4) ^ddd^ *P* < 0.001 versus THC (Tualang honey 200 mg/kg). (b) Thickness of endometrium of uterus in all experimental groups. BPA-induced reduction in thickness of the endometrium layer (PC group) was significantly prevented by concurrent treatment with Tualang honey (TH group). Data are expressed as Mean ± SEM. (1) ^aa^ *P* < 0.01 versus NC (negative control). (2) ^b^ *P* < 0.05, ^bb^ *P* < 0.01, and ^bbb^ *P* < 0.001 versus PC (BPA 10 mg/kg). (3) ^c^ *P* < 0.05 versus TH (Tualang honey 200 mg/kg + BPA 10 mg/kg). (4) ^ddd^ *P* < 0.001 versus THC (Tualang honey 200 mg/kg). (c) Thickness of myometrium of uterus in all experimental groups. BPA-induced reduction in the thickness of the myometrium layer (PC group) was significantly prevented by concurrent treatment with Tualang honey (TH group). Data are expressed as Mean ± SEM. (1) ^aa^ *P* < 0.01 versus NC (negative control). (2) ^bb^ *P* < 0.01 versus PC (BPA 10 mg/kg). (3) ^c^ *P* < 0.05 versus TH (Tualang honey 200 mg/kg + BPA 10 mg/kg). (4) ^dd^ *P* < 0.01 versus THC (Tualang honey 200 mg/kg).

**Figure 4:** Representative sections of uteri from all experimental groups (H&E, ×40). Normal histological appearance was observed in control group (NC group) ((A), (B), and (C)). Significant disruptive morphological changes were observed in BPA-exposed rats (PC group) ((D), (E), and (F)). The uterus of rat treated with Tualang honey alone (THC group) ((G), (H), and (I)) was comparable to the control group, while concurrent treatment of rats with BPA and Tualang honey (TH group) ((J), (K), and (L)) showed partial prevention of tissues damage from the toxic effect of BPA.

**Figure 5:** Representative sections of uteri showing the immunohistological localization of ER*α* in all experimental groups (×40). The most pronounced immunostaining intensity in both control ((C), (D)) (NC groups) and Tualang honey treated alone ((G), (H)) (THC groups) rats. Lower immunostaining intensity in BPA-exposed rats ((E), (F)) (PC group) was observed. Concurrent treatment with Tualang honey TH group ((I), (J)) also showed similar immunostaining intensity with these BPA-exposed rats.

**Figure 6:** Representative sections of uteri showing the immunohistological localization of ER*β* in all experimental groups (×40). The most pronounced immunostaining intensity was observed in BPA-exposed rats ((E), (F)) (PC group). Comparable immunostaining intensities were observed in NC ((C), (D)), THC ((G), (H)), and TH ((I), (J)) groups.

**Figure 7:** The lowest intensity of immunostaining was observed in BPA-exposed animals (PC group) ((E), (F)). However, higher intensity of color in stroma was noted with concurrent treatment with Tualang honey (TH group) ((I), (J)). Compared to the PC and TH groups, the highest and comparable immunostaining intensity were observed in NC group ((C), (D)) and THC group ((G), (H)).

**Figure 8:** (a) Quantitative real-time PCR of ER*α* in all experimental groups. ER*α* mRNA expression was significantly downregulated in the rats exposed to BPA (PC group) (4-fold) as compared to the control animals (NC group). However, the decline was reversed (3-fold) by concurrent treatment with Tualang honey (TH group). Data are expressed as Mean ± SEM. (1) ^a^ *P* < 0.05 and ^aa^ *P* < 0.01 versus NC (negative control). (2) ^b^ *P* < 0.05, ^bb^ *P* < 0.01, and ^bbb^ *P* < 0.001 versus PC (BPA 10 mg/kg). (3) ^c^ *P* < 0.05 and ^cc^ *P* < 0.01 versus TH (Tualang honey 200 mg/kg + BPA 10 mg/kg). (4) ^d^ *P* < 0.05, ^dd^ *P* < 0.01, and ^ddd^ *P* < 0.001 versus THC (Tualang honey 200 mg/kg). (b) Quantitative real-time PCR of ER*β* in all experimental groups. Compared to the control rats (NC group), the expression of ER*β* was significantly upregulated (1.4-fold) in BPA-exposed rats (PC group) and this is reduced to 1.1-fold by concurrent treatment of Tualang honey (TH group). Data are expressed as Mean ± SEM. (1) ^aaa^ *P* < 0.001 versus NC (negative control). (2) ^bbb^ *P* < 0.001 versus PC (BPA 10 mg/kg). (3) ^cc^ *P* < 0.01 and ^ccc^ *P* < 0.001 versus TH (Tualang honey 200 mg/kg + BPA 10 mg/kg). (4) ^ddd^ *P* < 0.001 versus THC (Tualang honey 200 mg/kg). (c) Quantitative real-time PCR of complement C3 in all experimental groups. BPA exposure (PC group) caused a significant downregulation of the amount of complement C3 mRNA (9-fold) as compared to the control rats (NC group). This effect was completely reversed by concurrent treatment with Tualang honey (TH group). Data are expressed as Mean ± SEM. (1) ^aaa^ *P* < 0.001 versus NC (negative control). (2) ^bbb^ *P* < 0.001 versus PC (BPA 10 mg/kg). (3) ^cc^ *P* < 0.01 and ^ccc^ *P* < 0.001 versus TH (Tualang honey 200 mg/kg + BPA 10 mg/kg). (4) ^ddd^ *P* < 0.001 versus THC (Tualang honey 200 mg/kg).

**Table 1:** Sequences of primers and references for TaqMan-PCR.

Gene	Forward primer	Reverse primer	References (accession number)
Estrogen receptor-*α*	5′-AAGCTGGCCTGACTCTGCAG-3′	5′-GCAGGTCATAGAGAGGCACGA-3′	Spreafico et al. [31] (X61098)

Estrogen receptor-*β*	5′-CTCTGTGTGAAGGCCATGAT-3′	5′-GGAGATACCACTCTTCGCAATC-3′	Kuiper et al. [32] (U57439)

Complement C3	5′-CTGTACGGCATAGGGATATCACG-3′	5′-ATGCTGGCCTGACCTTCAAGA-3′	Misumi et al. [33] (X52477)

**Table 2:** Body weight gain, uterine relative weight, malondialdehyde (MDA) level, and uterine histomorphometry parameters in all experimental groups.

Group	Body weight gain (g)	Uterine relative weight (wet weight/body weight)	Malondialdehyde (MDA) level (*μ*M/*μ* protein)	Height of luminal epithelial cells (*μ*m)	Thickness of endometrium (*μ*m)	Thickness of myometrium (*μ*m)
NC	78.88 ± 14.61	1.89 ± 0.12^bbb^	0.0037 ± 0.00026^bbb^	30.51 ± 1.37^bbb,c^	571.87 ± 19.14^bb^	299.18 ± 16.86^bb^
PC	99.25 ± 9.90	1.41 ± 0.04^aaa,c,d^	0.0074 ± 0.00053^aaa,c,ddd^	18.88 ± 0.81^aaa,cc,ddd^	486.74 ± 10.15^aa,cc,ddd^	228.39 ± 8.91^aa,c,dd^
THC	89.5 ± 10.64	1.83 ± 0.07^bb^	0.0036 ± 0.00089^bbb^	28.23 ± 0.48^a,bbb^	574.25 ± 19.45^bbb^	299.26 ± 9.92^bb^
TH	92.5 ± 4.62	1.73 ± 0.04^b^	0.0049 ± 0.00064^b^	26.86 ± 0.68^bbb^	546.30 ± 3.78^b^	284.51 ± 16.63^bb^

Data are expressed as Mean ± SEM.

(1) ^a^ *P* < 0.05 and ^aa^ *P* < 0.01 versus NC (negative control).

(2) ^b^ *P* < 0.05, ^bb^ *P* < 0.01, and ^bbb^ *P* < 0.001 versus PC (BPA 10 mg/kg).

(3) ^c^ *P* < 0.05 and ^cc^ *P* < 0.01 versus TH (Tualang honey 200 mg/kg + BPA 10 mg/kg).

(4) ^d^ *P* < 0.05, ^dd^ *P* < 0.01, and ^ddd^ *P* < 0.001 versus THC (Tualang honey 200 mg/kg).

## Abbreviations

BPA: Bisphenol A
OSCC: Oral squamous cell carcinomas
ER*α*: Estrogen receptor-alpha
ER*β*: Estrogen receptor-beta
MDA: Malondialdehyde
TBARS: Thiobarbituric Acid Reactive Substances
PBS: Phosphate buffered saline
BHT: Butylated hydroxytoluene
RNA: Ribonucleic acid
cDNA: Complementary deoxyribonucleic acid
PCR: Polymerase chain reaction
NC: Negative control group
PC: Positive control group
TH: Tualang honey + BPA group
THC: Tualang honey control.
